RETRACTED

# Assessment of Clinical Diagnostic Efficacy of Pulmonary Function Test Based on DBN-SVM of Pediatric Asthma and Cough Variant Asthma

**DOI:** 10.1155/2022/1182114

**Published:** 2022-03-31

**Authors:** Hanyi Li, Xinmei Zhang, Qijun Zhao, Xiang Bai, Shuying Wang

**Affiliations:** Department of Pediatric Respiratory, Gansu Provincial Maternity and Child-Care Hospital, Lanzhou City 730050, Gansu, China

## Abstract

The diagnosis of asthma depends on the unprejudiced proof of the varying airflow obstruction. The pulmonary function tests are carried out to evaluate the clinical value of different types of respiratory diseases in children or infants. This study is focused on the clinical evaluation of the pulmonary function tests in the diagnosis of pediatric asthma and cough variant asthma. A differential diagnosis method for chronic obstructive pulmonary disease (COPD) and asthma-COPD overlap with complementary diagnostic value is proposed. For the pulmonary function tests, the COPD gene dataset was selected and feature selection was performed using the DBN-SVM scoring method. For analysis and comparison, the differential diagnosis models were built using ROC curves for the accuracy of the deep belief network model and the support vector machine model. The sensitive features associated with COPD and ACO classification using the deep belief network model were found to be in good agreement with known clinical diagnostic strategies. The clinical diagnosis tests for pulmonary pediatric asthma and cough variant asthma were conducted on two groups of children, with both groups containing a basis of comparison. 80 cases of pediatric asthma and cough variant asthma were admitted from 2013 to 2014 and 80 cases of children with a healthy physical examination. The results of the two groups were compared. The results showed that the levels of FEV1, PEF, and FVC were significantly lower (*P* < 0.05), in healthy children, and FEV1/FVC%, RV, and RV/TCL% were significantly higher (*P* < 0.05) in children with asthma and cough variant asthma during acute exacerbation and chronic persistence. There were no statistically significant differences in the duration of clinical remission (*P* > 0.05). Thus, the study suggests that confirmed cases of the diagnosis of pediatric asthma and cough variant asthma by pulmonary function tests were significantly higher than those of conventional tests (*P* < 0.05). From this study, we can conclude that pulmonary function tests can accurately diagnose pediatric asthma and cough variant asthma, and also accurately reflect the development of the child's disease, which is of high clinical value.

## 1. Introduction

Asthma is a chronic lung disease that causes the airways to get narrow, which results in shortness of breath and chest infections. Asthma can be characterized by recurrent episodes of cough, dyspnea, and wheezing. A cough variant asthma is a specific type of asthma with chronic cough as the major clinical manifestation. Both asthma and cough variant asthma are common diseases of the pediatric respiratory system, through routine examination and auscultation, it is observed that there is a high probability of a poor or wrong diagnosis of the specificity of the clinical symptoms of the disease. [1]. Pulmonary function tests can objectively and effectively reflect the actual lung conditions and functional indicators of children and are of high value for the definitive diagnosis, observation of the course of the disease, and determination of its efficacy [2].

RETRACTED

There is a lack of awareness of energy detection. Children's organs are not fully developed and their immune systems are not fully constructed, which predisposes them to allergic diseases, such as asthma as well as cough variant asthma. Children with asthma and cough variant asthma do not have typical clinical symptoms after the onset of the disease and cannot be clearly diagnosed [3]. The clinical symptoms of some children with asthma and cough variant asthma are similar to those of other respiratory diseases, and the inability to make a clear diagnosis in time prevents the selection of an effective treatment plan, misses the best treatment time, and has a negative impact on the prognosis of patients [4]. A pulmonary function test is a noninvasive examination technique to detect the physiological functions of the respiratory system that can directly and accurately measure the physiological indicators of lung function and has the advantages of a shorter diagnostic process and higher accuracy [5]. Pulmonary function tests can detect airway abnormalities in the early stages of respiratory disorders and can help patients assess how far their sickness has progressed. In the diagnosis of pediatric asthma and cough variant asthma, the clinical symptoms are mainly chronic cough, while pulmonary function tests can effectively differentiate the diagnosis and distinguish it from lung infections. Bronchial asthma is more harmful to the physical and mental health of pediatric patients. The pathological basis is the hyperresponsiveness of the respiratory tract, while pulmonary function tests can objectively and accurately indicate the obstruction of the respiratory tract and also assess the severity of respiratory inflammation in children with asthma, providing strong evidence for the diagnosis of the disease [6]. According to some previous clinical studies, cough variant asthma is caused by chronic inflammation of the airways, which causes harm to the bronchial epithelium and exposure of the vagal nerve endings. Small localized airway constrictions in response to tiny stimuli that impact the terminal cough receptors, resulting in a cough reflex. Therefore there are no evident signs and symptoms of wheezing. [7]. In clinical diagnosis, pulmonary function measurements can effectively indicate the physiological and pathological status of the respiratory system and provide an effective diagnostic basis for pediatric asthma and cough variant asthma.

RETRACTED

Chronic obstructive pulmonary disease (COPD) and asthmalike obstructive airway disease (OAD) [8] are common chronic lung diseases that cause severe disease burden and affect the quality of life. Although COPD and asthma differ in inflammatory patterns, immune mechanisms, and degree of reversibility of airflow obstruction, a large number of patients with COPD and asthma exhibit similar clinical symptoms. Asthma usually presents with intermittent and reversible airway obstruction, whereas COPD is progressive and irreversible. The comorbidity of COPD and asthma is called asthma-chronic obstructive pulmonary disease (COPD) overlap (ACO) [9], and its prevalence increases with age [10]. Therefore, the diagnosis and treatment of ACO have become particularly important. Compared to patients with COPD or asthma alone, patients with asthma-COPD overlap have more frequent acute effects [11]. Chronic obstructive pulmonary disease, asthma, and ACO are all heterogeneous diseases with more similarities in etiology, pathological changes, and clinical manifestations. COPD and asthma are difficult to distinguish because certain symptoms are only part of the disease development process. There are more similar features, and there are no criteria to determine whether the corresponding treatment measures and prognosis are consistent, so how to distinguish ACO from COPD alone is a hot topic in respiratory research. Although studies have shown that COPD is statistically different from asthma-COPD overlap in terms of lung function, clinical features, spirometry, chest CT scan, 6MWD, SGRQ, etc., these features cannot be used alone as a basis for classifying patients with asthma-COPD overlap (ACO) and COPD [12].

In this paper, we hypothesize that there are potential associations in the original clinical features related to disease diagnosis, and that such potential associations can build a robust model to provide computerized clinical decision support. Deep learning methods can discover potential correlations in high-dimensional data, and deep belief networks (DBNs) are one of the most successful structures in deep learning methods, and their good feature extraction capabilities are well demonstrated in both image and speech recognition [13]. DBNs are highly complex nonlinear feature extractors. Each layer of its hidden unit can learn and capture higher-level features from the original input data [14]. Therefore, in this paper, we use a large number of clinical data samples to construct a differential diagnosis model of COPD and ACO using the DBNs algorithm and support vector machine algorithm to provide a reference for clinical diagnosis.

RETRACTED

The following paper is organized as follows: deep confidence network algorithms are discussed in Section 2. After that, the related work is discussed in Section 3. It is followed by the case study of the paper in Section 4. Then results are presented in Section 5. Lastly, the discussion and conclusions have been explained in Section 6 and 7, respectively.

## 2. Deep Confidence Network Algorithm

The effectiveness and efficacy of chronic pulmonary disorders are studied using a deep trust network. Different algorithms, such as the restricted Boltzman machine and the DBM training procedure for developing structures to understand deep learning, have been explored in this section.

### 2.1. Restricted Boltzmann Machine (RBM)

The depth confidence network is composed of multiple RBMs stacked. The RBM is composed of visible layer *V* and hidden layer *h*. The neurons in visible layer *V* and hidden layer *h* are linked, but the neurons in the same layer are independent of one another. The neuron states of visible layer *V* and hidden layer *h* are represented by {0, 1} for activated and inactive states. RBM constructs the hidden layer through the connection weight *w*_*ij*_ of each neuron between the visible layer *V* and the hidden layer *h*. The information extracted by the hidden layer *h* can be regarded as the characteristics of the input visible layer *V* data. The structure of RBM is shown in Figure 1.

The visible layer neurons are represented as *v*={*v*_1_, *v*_2_,…, *v*_*n*_}, the hidden layer neurons are represented as *h*={*h*_1_, *h*_2_,…, *h*_*m*_}, and the energy function of RBM is represented as

(1) $$\begin{array}{c} E\left(v,h\right)=-\sum_{i=1}^{n}a_{i}v_{i}-\sum_{j=1}^{m}b_{j}h_{j}-\sum_{i=1}^{n}\sum_{j=1}^{m}w_{ij}v_{i}h_{j}, \end{array}$$

where *a*_*i*_ is the bias of neurons in the visible layer, *b*_*j*_ is the bias of hidden layer neurons, and *w*_*ij*_ is the weight of neuron connection.

The joint probability distribution function between the visible layer and the hidden layer is expressed as

(2) $$\begin{array}{c} P\left(v,h\right)=\frac{1}{\sum_{i=1}^{m}\sum_{j=1}^{n}e^{-E\left(v,h\right)}}e^{E\left(v,h\right)}. \end{array}$$

The conditional distribution probability of visible layer *V* and hidden layer *h* can be expressed as

(3) $$\begin{array}{c} p\left(h_{j}=1|v\right)=\mathrm{sigmoid}\left(b_{j}+\sum_{i=1}^{n}w_{ij}v_{i}\right),\\ p\left(v_{i}=1|h\right)=\mathrm{sigmoid}\left(a_{i}+\sum_{i=1}^{m}w_{ij}v_{i}\right). \end{array}$$

By using the contrast divergence (CD) algorithm, the update of weight and offset can be expressed as

(4) $$\begin{array}{c} \Delta w_{ij}=\eta \left({\langle v_{i}h_{j}\rangle }_{\text{data}}-{\langle v_{i}h_{j}\rangle }_{\text{recon}}\right), \end{array}$$

(5) $$\begin{array}{c} \Delta a_{i}=\eta \left({\langle v_{i}\rangle }_{\text{data}}-{\langle v_{i}\rangle }_{\text{recon}}\right), \end{array}$$

(6) $$\begin{array}{c} \Delta b_{j}=\eta \left({\langle h_{j}\rangle }_{\text{data}}-{\langle h_{j}\rangle }_{\text{recon}}\right), \end{array}$$

where *η* is the learning rate. The RBM can be updated and optimized through equations (4) to (6).

RETRACTED

### 2.2. DBN Training Process

The hidden layer of the upper RBM is stacked as the visible layer of the lower RBM to form a deep confidence network [15]. The input data is inserted from the visible layer of the lowest RBM. The unsupervised learning of all RBMs in the DBN is completed from bottom to top according to the above RBM training process. The RBM output feature of the top layer is the extracted feature of the input data. According to the data characteristics, the top RBM output can pass through the Softmax classifier to form a data classification label. The label is compared with the original data label and calculated to form a modeling error. The RBM connection weight in the DBN is supervised and optimized through the error backpropagation algorithm [16].

To summarize, DBN training is a comprehensive process of unsupervised and supervised learning that leads to a more accurate extraction of data features.

### 2.3. Least Squares Support Vector Machine Health State Partition Algorithm

In this paper, the least squares support vector machine is used to divide the health state of the feature parameters extracted by the DBN model. The feature parameters obtained by the DBN model are the input parameters. After mapping the LSSVM kernel function to the high-dimensional space, it is divided. The high-dimensional hyperplane is used to classify the different feature parameters.

The support vector machine algorithm transforms the classification problem into an optimization problem, uses the principle of structural risk minimization, and selects the loss function as the quadratic term of the error. For the sample set (*x*_*i*_, *y*_*i*_)_*i*=1_^*N*^

(7) $$\begin{array}{c} \left\{\begin{array}{c} \min J\left(\omega ,\xi \right)=\frac{1}{2}\omega^{\text{T}}\omega +\frac{1}{2}c{\overset{N}{\underset{i=1}{\sum }}\xi }_{i}^{2},\\ s.t.\;y_{i}=\omega^{\text{T}}\varphi \left(x_{i}\right)+b+\xi_{i}. \end{array}\right) \end{array}$$

In support vector machine algorithm, a kernel function is usually used to represent the mapping from sample space to high-dimensional space, which can be expressed as

(8) $$\begin{array}{c} K_{ij}\left(x_{i},x_{j}\right)=\varphi {\left(x_{i}\right)}^{T}.\varphi \left(x_{j}\right). \end{array}$$

The above equation is solved by the Lagrange method, and the optimization problem can be expressed as

(9) $$\begin{array}{c} \left[\begin{array}{cc} 0 & 1\\ 1 & \Phi +V_{c} \end{array}\right]\left[\begin{array}{c} b\\ \alpha \end{array}\right]=\left[\begin{array}{c} 0\\ y \end{array}\right], \end{array}$$

where the estimation of

**y**=[*y*_1_, *y*_2_,…,*y*_*N*_]^*T*^; *α*=[*α*_1_, *α*_2_,…,*α*_*N*_]^*T*^, **V**_c_=diag{1/*c*}; Φ=[*K*_*ij*_*|i*, *j*=1,2,…,*N*]^*T*^ Sample classification labels can be expressed as

(10) $$\begin{array}{c} y^{*}\left(x\right)=\sum_{i=1}^{N}\alpha_{i}K\left(x,x_{i}\right)+b. \end{array}$$

Gaussian radial basis function (RBF) is selected as

(11) $$\begin{array}{c} K\left(x,x_{i}\right)=e^{-{\left\|x-x_{i}\right\|}^{2}/\sigma^{2}}, \end{array}$$

where unknown parameters *c* and *σ* it is obtained by the grid search and crossvalidation method in reference [17].

RETRACTED

An SVM is a machine learning algorithm based on different kernels. This study uses four kinds of kernels. According to the two evaluation indexes of model classification accuracy and ROC curve, the appropriate kernels are selected to construct the support vector machine model.

DBNs are the most common type of architecture in deep learning. In order to find DBNs with suitable structures in a practical problem, the number of hidden layer layers and the number of nodes in each hidden layer must be determined. The number of visible layer nodes is equal to the number of input features. In this paper, three 3-layer DBNs with different structures are constructed, and the number of nodes in the hidden layers is 50–50, 100–50, and 100–100, respectively. The appropriate structures are chosen to construct DBN models according to the classification accuracy of the model.

The training samples are used to construct the support vector machine model and the deep belief network model, and then the prediction samples are used to test the performance of the two models. Finally, the two models are compared by model classification accuracy, ROC curve, sensitivity, and specificity. MATLAB r2016a was used to process and statistically analyze the data. The counting variables were represented by $\bar{x}\pm \text{SD}$ and analyzed by *t*-test; Categorical variables were analyzed by *x*^2^ test. The subject operating characteristic curve (ROC curve) analysis method was used to calculate the sensitivity, specificity, and accuracy to evaluate the prediction performance of the model.

RETRACTED

## 3. Related Work

The data for this study were obtained from the COPD gene database constructed by the National Heart, Lung, and Blood Institute (NHLBI). Based on the given data, the study subjects were divided into a COPD-only group (2,919 cases) and an asthma-COPD overlap (ACO) group (1,116 cases).

The total number of data items for the participating subjects was 361, including demographic information, medical history, clinical assessment scales, tests, and physical examination [18].

The COPD gene dataset used in this study contains 361 features, and 320 features remain after removing the features with large data missing. The dataset was randomly divided into 10 parts using the 10-fold cross-validation (10FCV) method, of which 90% were used as training samples and 10% as prediction samples. To improve the model's accuracy for disease classification, features were chosen using the Fisher score method, which calculates a feature's Fisher score value to indicate how sensitive the feature is to the classification result [19]. Four subsets of features were selected from the top 320, 240, 120, and 80 features according to the score value, and the appropriate subset of features was selected according to the accuracy of the model. The research method has the following 2 main mathematical models.

## 4. Case Study

Eighty children with asthma and cough variant asthma were admitted to our hospital from January 2014 to December 2014 were selected, and all of them met the relevant diagnostic criteria in the “Guidelines for the prevention and treatment of bronchial asthma (definition, diagnosis, treatment, and education and management program of bronchial asthma)” formulated by the Asthma Group of the Chinese Medical Association's Respiratory Diseases Branch in 2003 [20]. The control group consisted of another 80 healthy children who had been immunized in our hospital, and the lung function test results of the children examined in both groups were statistically compared. In both groups, serious organic pathologies such as heart, liver, and kidney diseases as well as hereditary diseases were excluded. The general data of gender and age of the children in both groups were statistically analyzed, and there was no significant difference between the groups in the indexes (*P* > 0.05), which was suitable for the controlled study.

RETRACTED

The results of pulmonary function tests in the two groups of children are shown in Table 1, and the FEV1, PEF, and FVC of the children in the observation group were significantly lower (*P* < 0.05) and FEV1/FVC%, RV, and RV/TCL% were significantly higher (*P* < 0.05) than those in the control group during the acute exacerbation and chronic persistence (*P* > 0.05).

The accurate diagnostic value of conventional and pulmonary function tests for pediatric asthma and cough variant asthma is shown in Table 2. The diagnostic rates of pulmonary function test for typical asthma and cough variant asthma were significantly higher than those of conventional tests (*P* < 0.05).

## 5. Results and Analysis

In this section, the results obtained from the computational model through analysis have been discussed. The details of the results are as follows:

### 5.1. Feature Selection and Model Parameter Selection

After feature selection, the classification accuracy results of the DBNs model are shown in Table 3. The highest accuracy was obtained by using the top 160 features of the Fisher score as the input of the DBNs model. These 160 features were selected as the input features of the SVM model and DBNs model.  Figure 2 shows the classification accuracy of DBN models with 3 hidden cell structures for 2 diseases at different iterations. This shows the classification accuracy of DBN models with different structures. Therefore, the 50–50 hidden cell structure was chosen to build the final DBNs model.

### 5.2. Model Construction Results

The accuracy, sensitivity (indicating the proportion of COPD pairs classified in the prediction sample), and specificity (indicating the proportion of ACO pairs classified in the prediction sample) of the model were calculated by using the training samples to construct the support vector machine model and the deep belief network model, as shown in Table 4. The ROC curves were obtained (Figure 3). The accuracy of DNBs was the highest (93.56%), while the accuracy of the four support vector machine algorithms with different kernels did not reach 90%. Among the prediction samples, the highest COPD identification rate (sensitive) is for the DBNs model (95.21%), while the highest SVM model is 89.73%, and the highest ACO identification rate (specificity) is still for the DBNs model (89.29%), corresponding to the highest SVM model (74.11%). Figure 3 depicts the subject operating characteristic curves (ROC) of the five models, and the ROC curve of the DBNs model is closest to the upper left corner and completely above the ROC curves of the support vector machine models with four different kernels, indicating that the DBNs model outperforms the support vector machine model in classification.

RETRACTED

### 5.3. Feature Importance Ranking

The COPD-gene database contains data on various clinical, physiological, imaging, and biological aspects of the study subjects [21]. The top ten sensitivity features were calculated using the DBNs model and were derived from five different scales in the COPD-gene database: the smoking status scale, the CT impact outcome scale, the clinical diagnosis scale, the health status scale, and the lung function scale. The 10 features included 5 categories of indicators, 1 of which belonged to smoking status (duration of smoking), 3 to CT imaging results (TLC_CT, Slicer_IntensityMean_Ex, and Vida_15perc_Exp), 2 clinical diagnoses (Bronch Dx By Dr, Sleep Ap Still-Hav), 2 health status (destalked, SF36 _ PF _ *t* _score), and 2 lung function scales.), and 2 in pulmonary function (pre_FEV1, pre_FVC).

Applying statistical analysis with the Pearson *x*^2^ test for categorical variables and *t*-test for numerical variables, 10 characteristics were statistically significantly different in COPD and ACO with *P*-values less than 0.05. By hypothesis testing, it was found that these 10 sensitive characteristics had different distributions, as shown in Table 5.

## 6. Discussion

In this paper, we propose a new method for differential diagnosis of ACO and COPD using DBNs for the first time and compare it with the support vector machine model in terms of accuracy, sensitivity, specificity, and ROC curves. The results show that the DBNs model has better classification than the support vector machine model, demonstrating that the DBNs model can learn essential features from the dataset.

With the exception of the traditional clinical importance of risk factor analysis, the importance magnitude of DBN model predictor variables reflect the extent to which the corresponding indicators contribute to the model in distinguishing the two diseases, i.e., the more highly ranked predictor variables contribute to the model's use in distinguishing the two diseases. The problem of high-dimensional data is encountered in numerous applications of machine learning and data mining [16]. The features with high Fisher scores among the 320 features in this paper were selected as the input vector for the DBNs model, and the results showed that the DBNs model built after filtering features using Fisher scores could achieve higher accuracy.

High levels of multivariate features may be associated with certain characteristics of a disease and can be used to build a sophisticated data-driven model to classify the disease. The parametric DBNs model developed in this paper identifies sensitive factors that are consistent with clinical a priori knowledge. In evaluating the strengths and weaknesses of this paper, DBNs were compared with SVMs. For this binary classification problem, DBNs have an accuracy of 93.56%, sensitivity of 95.21%, and specificity of 89.29%, while the highest accuracy of four typical support vector machine models is 85.40%, sensitivity of 89.73%, and specificity of 74.11%, indicating that compared with support vector machines, a traditional machine learning model, DBNs have better classification ability [22].

RETRACTED

The DBNs model was used to identify sensitive features associated with COPD disease. The top 10 variables in the predictive importance of the DBN model output included subjects' CT imaging findings, clinical diagnosis, health status, smoking status, and lung function. These functions were strongly associated with the etiology of COPD and ACO, indicating that the sensitive features identified by the DBNs model are consistent with the main factors in the current clinical diagnosis of ACO factors are consistent. In addition, the results of the descriptive analysis showed that there were statistical differences between COPD and ACO for the first 10 sensitive features. The features extracted by the DBNs model can effectively distinguish between these two diseases with similar symptoms. The top ten sensitive features identified in this paper suggest that internal medicine physicians should consider not only biochemical tests, laboratory tests, and imaging data, but also epidemiological factors, health status, and even personal habits when diagnosing patients with COPD or ACO.

## 7. Conclusions

The findings suggest that a deep belief network model using multiple types of features from lung function, disease status, demographic data, and health status data can effectively distinguish COPD from ACO. Sensitive features associated with COPD and ACO classification are in good agreement with clinical diagnostic strategies and contribute to a better understanding of COPD and asthma in children, due to the overlapping etiology and symptoms of COPD. The differential diagnosis of COPD and ACO is important because these two diseases differ in terms of treatment, morbidity, and mortality. Deep learning methods can be used to improve the standard of living and potential patient survival by preventing and treating COPD and ACO. The DBNs model developed in this paper can achieve high judgment accuracy, indicating that the deep learning model is expected to be a diagnostic decision aid.

## Figures and Tables

**Figure 1:** RBM structure diagram.

**Figure 2:** Classification accuracy of DBNs models with different structural hidden units for COPD and ACO with a different number of iterations.

RETRACTED

**Figure 3:** ROC curves of DBNs and SVMs of 4 kernels.

**Table 1:** Results of pulmonary function tests in children with asthma and cough variant asthma and healthy children ($\bar{x}\pm s$,*n* = 80).

Group		FEV1(L)	FEV1/FVC%	PEF(L/S)	RV/TCL%	RV/TCL%	FVC(L)
	Chronic duration	87.54 ± 10.21	78.27 ± 7.18	78.89 ± 8.67	3.09 ± 0.68	47.15 ± 10.17	73.58 ± 5.81
	Clinical remission	91.89 ± 9.42	77.29 ± 2.62	81.47 ± 9.53	2.48 ± 0.52	40.92 ± 11.79	82.16 ± 8.25
Control group		92.64 ± 10.73	80.15 ± 5.90	84.54 ± 8.39	2.09 ± 0.28	97.99 ± 7.85	85.47 ± 11.24

**Table 2:** Comparison of the diagnostic accuracy of conventional examination and pulmonary function tests in children in the observation group *n*(%).

Method	Typical asthma (*n* = 48)		Cough variant asthma (*n* = 32)	
	Diagnostic rate	Misdiagnosis rate	Diagnostic rate	Misdiagnosis rate
Routine inspection	38(79.17)	10(20.83)	15(46.88)	17(53.12)
Pulmonary function test	47(97.92)	1(2.08)	30.(93.75)	2(6.25)
*x* ^2^	−1.6318	1.6318	−2.5154	2.5158
*P* value	<0.05	<0.05	<0.05	<0.05

**Table 3:** Accuracy of DBNs models after feature selection.

Number of features	Accuracy of DBNs model/%
320	81.05
240	87.10
160	93.56
80	90.45

**Table 4:** Classification accuracy, sensitivity, and specificity of DBNs and SVMs with 4 different kernels.

Model	Accuracy%	Sensitivity%	Specificity%
SVM-linear	82.43	86.99	70.54
SVM-polynomial	85.40	89.73	74.11
SVM-radial-basis function	82.92	88.36	68.14
SVM-sigmoid	73.27	75.34	67.86
DBNs	93.56	95.21	89.29

**Table 5:** Distribution of the top 10 relatively important characteristics of COPD and ACO classification.

Serial number	Variable	COPD(*n* = 2919)	ACO(*n* = 1116)	*P* value
1	TLC_CT	6.15 ± 1.44	5.85 ± 1.45	<0.001
2	Bronchdxby Dr (yes)	12.05(41.28)	709(65.53)	<0.001
3	Slicer intensity mean_Ex	−773.96 ± 60.65	−779.38 ± 58.25	0.010
4	Destalked	1264.24 ± 404.61	1174.38 ± 407.30	<0.001
5	Vida_15perc_Exp	-903.46 ± 48.25	908.43 ± 47.15	0.018
6	SF36 _ PF _ *t* _score	39.56 ± 12.1	34.47 ± 12.09	<0.001
7	Sleep ap Still-Hav(Yes)	370(12.68)	214(19.18)	<0.001
8	Duration smoking	40.54 ± 9.51	37.42 ± 9.82	<0.001
9	pre_FEV1	1.65 ± 0.62	1.36 ± 0.48	<0.001
10	pre_FVC	3.01 ± 1.03	2.36 ± 0.97	<0.001

## Data Availability

The datasets used and analyzed during the current study are available from the corresponding author upon reasonable request.
